The article "miR-484 suppresses proliferation and epithelial–mesenchymal transition by targeting ZEB1 and SMAD2 in cervical cancer cells" was retracted in 2021. Reasons: duplicated images; unreliable results or conclusions; concerns about the data.

# miR-484 suppresses proliferation and epithelial–mesenchymal transition by targeting ZEB1 and SMAD2 in cervical cancer cells

**DOI:** 10.1186/s12935-017-0407-9

**Published:** 2017-03-07

**Authors:** Yang Hu, Hong Xie, Yankun Liu, Weiying Liu, Min Liu, Hua Tang

**Affiliations:** Tianjin Life Science Research Center and Department of Pathogen Biology, School of Basic Medical Sciences, Tianjin Medical University, 22 Qi-Xiang-Tai Road, Tianjin, 300070 China

**Keywords:** miR-484, SMAD2, ZEB1, EMT, Cervical cancer

## Abstract

**Background:**

MicroRNAs (miRNAs) play important roles in cancer initiation and development. Epithelial–mesenchymal transition (EMT) is a form of cellular plasticity that is critical for embryonic development and metastasis. The purpose of the study was to determine the function and mechanism of miR-484 in initiation and development of cervical cancer (CC).

**Methods:**

We determined the expression levels of miR-484 in cervical cancer tissues and cell lines with RT-qPCR. Prediction algorithms and EGFP reporter assay were performed to evaluate the targets for miR-484. MTT assay, colony formation assay, flow cytometric analysis, transwell cell migration and invasion assays, and detection of EMT markers were employed to investigate the roles of miR-484 and the targets in regulation of cell proliferation and EMT process. We also used rescue experiments to confirm the effect of miR-484 on CC cells through directly regulating the expression of its targets.

**Results:**

Firstly we found miR-484 was down-regulated in cervical cancer tissues and cell lines compared with their matched non-cancerous tissues or normal cervical keratinocytes cells. Further studies revealed that overexpression of miR-484 suppressed the cell proliferation, while exacerbates apoptosis. Besides, miR-484 suppressed cellular migration, invasion and EMT process of CC cells. EGFP reporter assay showed that miR-484 binds to ZEB1 and SMAD2 3′UTR region and reduced their expression. The expression of miR-484 had reverse correlation with SMAD2/ZEB1, and SMAD2/ZEB1 had positive correlation with each other in cervical cancer tissues and cell lines. Furthermore, the ectopic expression of ZEB1 or SMAD2 could rescue the malignancies suppressed by miR-484, suggesting that miR-484 down-regulates ZEB1 and SMAD2 to repress tumorigenic activities.

**Conclusion:**

We found miR-484 inhibits cell proliferation and the EMT process by targeting both ZEB1 and SMAD2 genes and functions as a tumor suppressor, which may served as potential biomarkers for cervical cancer.

## Background

Cervical cancer (CC) is the fourth leading cause among cancer-related deaths in women, and due to delayed initial screening, it mainly occurs in developing countries and causes about 265,000 deaths every year worldwide [1]. Nowadays, advances in CC therapies have improved treatment outcomes, while the prognosis remains limited and ineffective and a great number of patients died of metastasis. Although human papilloma virus (HPV) is the major risk factor for CC [2, 3], independent alterations in tumour suppressor genes and oncogenes are essential for the development of these cancers as well [4, 5]. Therefore, it’s crucial to identify specific molecules and markers that contribute to understanding cervical carcinogenesis and ascertaining diagnostic and treatment strategies. Recently, researchers have focused on the effect of miRNAs on CC and a lot of miRNAs were found to play great importance in the initiation and development of CC [6–8].

The article "miR-484 suppresses proliferation and epithelial–mesenchymal transition by targeting ZEB1 and SMAD2 in cervical cancer cells" was retracted in 2021. Reasons: duplicated images; unreliable results or conclusions; concerns about the data.

MicroRNAs are a class of 18-25-nucleotide, highly conserved non-coding RNAs that post-transcriptionally regulate gene expression by binding to their 3′UTRs and regulate a wide range of physiological and pathological processes including cell differentiation, proliferation, apoptosis, invasion and migration [9–12]. In addition, growing evidences indicate that miRNAs are aberrantly expressed in human cancers and may function as tumor suppressors or oncogenes [13]. miR-484 was located on chr6. The expressions and functions of miR-484 in cancers were little. Although Yang et al. [14] reported that miR-484 was overexpressed in premalignant lesions of hepatocellular carcinoma (HCC), and can promote hepatocyte transformation and hepatoma development in two hepatocyte orthotopic transplantation models. Until now, the role and mechanism of miR-484 in CC cells are not clear.

Epithelial–mesenchymal transition (EMT) is an essential requirement for cancer invasion and metastasis [15–17]. The transcription factors Snail, Slug, Twist, zinc finger E-box-binding homeobox (ZEB) play vital role in initiation of EMT process. Recent reports have showed that the miR-200 family and other miRNAs regulate EMT through targeting these transcription factors [18–20]. ZEB family factors (ZEB1 and ZEB2) are transcriptional repressors that comprise two widely separated clusters of C2H2-type zinc fingers which bind to paired CAGGTA/G E-box-like promoter elements. These factors promote EMT by repressing expression E-cadherin [21–23] and are important intracellular mediators of TGFβ-induced EMT. Over the past few years, ZEB1 has increasingly been considered as an important contributor to the process of malignancies including endometrioid cancer [24], breast cancer [25], lung adenocarcinomas [26] as well as cervical cancer [27]. On the one hand, it has been shown that miRNAs, such as the miR-200 family can directly bind to 3′UTR of the ZEB mRNA to down-regulate its expression and influence epithelial differentiation [28, 29]. On the other hand, it has been revealed that SMAD proteins directly act with the promoter of the ZEB factor and indirectly regulates establishment and maintenance of EMT [30, 31].

The article "miR-484 suppresses proliferation and epithelial–mesenchymal transition by targeting ZEB1 and SMAD2 in cervical cancer cells" was retracted in 2021. Reasons: duplicated images; unreliable results or conclusions; concerns about the data.

In this report, we demonstrated that miR-484 is down-regulated in cervical cancer tissues and cell lines, and overexpression of miR-484 inhibits cell proliferation, cell viability and exacerbates apoptosis, suppresses cell migration, invasion and EMT process of CC cells as well. Moreover, miR-484 was validated to directly bind to the 3′UTR of the ZEB1 and SMAD2 transcript, inhibiting their expression in CC cells. We also found that SMAD2 is an upstream regulator of ZEB1. Therefore, miR-484 regulated EMT process through both directly and indirectly targeting ZEB1. Collectively, our present work provides the first evidence that miR-484 down-regulates ZEB1 and SMAD2 expression to repress malignant properties in CC cells. The findings may provide insights into the mechanisms underlying carcinogenesis and potential biomarkers for cervical cancer.

## Methods

### Human cervical cancer tissue specimens and cell lines

Fifteen CC tissues and the paired adjacent non-tumor cervical tissues were obtained from the cancer center of Sun Yat-sen University. The diagnose was evaluated by pathological analysis. Written informed consent was obtained from each patient and ethics approval for this work was granted by the Ethics Committee of Sun Yat-Sen University. The cervical samples were classified by pathologists. The human CC cell lines HeLa, Caski and ME-180 were maintained in RPMI-1640 medium. C33A, SiHa and SW756 were maintained in MEM-α medium according to Ref. [32]. Primary cultures of normal cervical keratinocytes (NCx) were obtained from hysterectomy specimens removed for non-neoplastic disease unrelated to the cervix. Cell culture and determination of growth rates were according to Ref. [33]. All the cells were maintained in a humidified incubator with 5% carbon dioxide (CO_2_) at 37 °C.

### Vector construction

To over-express miR-484, the primary miR-484 fragment was amplified from genomic DNA and cloned into pcDNA3 vector between *Bam*HI and *Eco*RI sites. To block the function of miR-484, we purchased the 2′-*O*-methyl-modified antisense oligonucleotide of miR-484 (ASO-miR-484) and the scramble control oligonucleotides (ASO-NC) from the GenePharma (Shanghai, China).

The gene encoding ZEB1/SMAD2 was amplified from the cDNA of HeLa cells, and the product was cloned into pcDNA3-Flag vector between *Eco*RI and *Xho*I sites. The shRNA for knocking down SMAD2 and ZEB1 were synthesized from GenePharma (Shanghai, China) and were annealed and cloned into pSilencer 2.1-neo vector (Ambion) between *Bam*HI and *Hin*dIII sites.

The article "miR-484 suppresses proliferation and epithelial–mesenchymal transition by targeting ZEB1 and SMAD2 in cervical cancer cells" was retracted in 2021. Reasons: duplicated images; unreliable results or conclusions; concerns about the data.

The 3′UTR of ZEB1/SMAD2 (containing the predicted binding sites for miR-484) was amplified from the cDNA of HeLa cells and then was cloned into pcDNA3-EGFP vector between the *Bam*HI and *Eco*RI sites (downstream of EGFP). The mutant 3′UTR of ZEB1/SMAD2 (five nucleotides were mutated in the miR-484 binding sites) was amplified from the construct (pcDNA3-EGFP/ZEB1 or pcDNA3-EGFP/SMAD2 3′UTR). All of the primers for PCR amplification and all the oligonucleotides for annealing are listed in Table 1.

**Table 1:** The oligonucleotides and primers used in this study

Name	Sequence (5′–3′)
Pri-miR-484-forward	CGACGGATCCAAGCGCACCCTTCACTTC
Pri-miR-484-reverse	GCTCGAATTCCGCTTCAAGGTTCCTTTCG
ASO-miR-484	AUCGGGAGGGGACUGAGCCUGA
ASO-NC	CAGUACUUUUGUGUAGUACAA
SMAD2-forward	GCGGAATTCAACATGTCGTCCATCTTGCCATTC
SMAD2-reverse	CCAGCTCGAGTTATGACATGCTTGAGCAACG
ZEB1-forward	GCGGATCCGCGGATGGCCCCAGGTGTAAG
ZEB1-reverse	GACGCCTCGAGTTAGGCTTCATTTGTCTTTTCTTC
SMAD2-3′UTR-S	GATCCTTTCTAGTATCTTACAGCCTGATAAGCTTG
SMAD2-3′UTR-AS	AATTCAAGCTTATCAGGCTGTAAGATACTAGAAAG
ZEB1-3′UTR-S	GATCCTTCTGGAGAGGTCAGAGTTGACAAGCTTG
ZEB1-3′UTR-AS	AATTCAAGCTTGTCAACTCTGACCTCTCCAGAAG
SMAD2-3′UTRmut-S	GATCCTTTCTAGTATCTTACCGAGCTATAAGCTTG
SMAD2-3′UTRmut-AS	AATTCAAGCTTATAGCTCGGTAAGATACTAGAAAG
ZEB1-3′UTRmut-S	GATCCTTCTGGAGAGGTCATCTAACTACAAGCTTG
ZEB1-3′UTRmut-AS	AATTCAAGCTTGTAGTTAGATGACCTCTCCAGAAG
miR-484-RT primer	GTCGTATCCAGTGCAGGGTCCGAGGTGCACTGGATACGACATCGGGAG
miR-484-forward	TGCAGTCAGGCTCAGTCCCC
U6-RT primer	GTCGTATCCAGTGCAGGGTCCGAGGTATTCGCACTGGATACGACAAAATATGGAAC
U6-forward	TGCGGGTGCTCGCTTCGGCAGC
Reverse primer	CCAGTGCAGGGTCCGAGGT
qPCR-actin-forward	CGTGACATTAAGGAGAAGCTG
qPCR-actin-reverse	CTAGAAGCATTTGCGGTGGAC
qPCR-ZEB1-forward	TAAAGTGGCGGTAGATGGTA
qPCR-ZEB1-reverse	ACTGTTTGTAGCGACTGGATT
qPCR-FN1-forward	CAGTGGGAGACCTCGAGAAG
qPCR-FN1-reverse	TCCCTCGGAACATCAGAAAC
qPCR-Snail-forward	TTCTCTAGGCCCTGGCTGC
qPCR-Snail-reverse	TACTTCTTGACATCTGAGTGGGTCTG
qPCR-Twist-forward	GCAAGAAGTCGAGCGAAGAT
qPCR-Twist-reverse	GCTCTGCAGCTCCTCGAA

### Prediction of miRNA targets

miR-484 predicted targets were retrieved from TargetScan (http://genes.mit.edu/tscan/targetscanS.html), miRecords (http://c1.accurascience.com/miRecords/) and PITA (https://genie.weizmann.ac.il/pubs/mir07/) and the binding site predictions were performed using RNAhybrid (http://bibiserv.techfak.uni-bielefeld.de/rnahybrid/).

### Cell transfection

Transient transfection was performed in antibiotic-free Opti-MEM medium (Invitrogen) with the Lipofectamine 2000 reagent (Invitrogen, Carlsbad, CA) following the manufacturer’s protocol.

The article "miR-484 suppresses proliferation and epithelial–mesenchymal transition by targeting ZEB1 and SMAD2 in cervical cancer cells" was retracted in 2021. Reasons: duplicated images; unreliable results or conclusions; concerns about the data.

### RNA isolation and reverse transcription quantity (RT-qPCR)

Extraction of total RNA from cells was performed using the TRIzol reagent (Invitrogen, CA) following the manufacturer’s instructions. Expression of mature miRNAs and mRNAs were quantified by RT-qPCR using the SYBR Premix Ex TaqTM (Promega, Madison, WI). The concentration of RNA were measured with a NanoDrop 2000 spectrophotometer (Thermo Fisher Scientific, Waltham, MA, USA) and stored at −80 °C for further use. Special stem-loop primers were used for the miRNA reverse transcription (RT) reaction, and U6 small nuclear B noncoding RNA (RNU6B) was used as the endogenous control to normalize the level of miRNA. The oligo (dT) primer was used for the RT reaction for gene expression. β-actin was used as the endogenous control to normalize the level of genes. All analyses were performed in triplicate and reported as 2^−ΔΔCt^. The primers for RT and PCR are provided in Table 1.

### Fluorescent reporter assays

To identify the direct target relationship between miR-484 and the 3′UTR of ZEB1/SMAD2 mRNA, the CC cells were cotransfected with pcDNA3/pri-miR-484 or ASO-miR-484 and the 3′UTR of ZEB1/SMAD2 or the mutant 3′UTR of ZEB1/SMAD2 in 48-well plates. The vector pDsRed2-N1 (Clontech, Mountain View, CA) expressing RFP (red fluorescent protein) was transfected together with the above plasmids and used as an internal control standard. 48 h after transfection, the cells were lysed by RIPA buffer and fluorescence intensities of EGFP and RFP were detected with an F-4500 fluorescence spectrophotometer (Hitachi, Tokyo, Japan).

### Cell viability assay and colony formation assay

The cell viability of CC cells was evaluated by the 3-(4,5-dimethylthiazol-2-yl)-2,5-diphenyl-tetrazolium bromide (MTT) assay. The absorbance was determined at 570 nm (A570) (Bio-Tek Instruments, Winooski, VT, USA) after CC cells transfection for 24, 48 and 72 h. The details of methods were according to Ref. [34].

For colony formation assay, the cells were seeded into 12-well plates at a density of 300 HeLa or 400 C33A per well at post-transfection 24 h. Change medium every 3 days. After 11 or 13 days, the cells were stained with crystal violet, and colonies including more than 50 cells were counted. The average number was used to evaluate the formation ability.

### Cell cycle analysis and apoptosis assay by flow cytometry

Cell cycle analysis and apoptosis assay was according to Refs. [6] and [35] respectively.

### Cell migration and invasion assays

The migration and invasion were analyzed by 24-well Boyden chambers with an 8-μm pore size polycarbonate membrane (Corning, Cambridge, MA). Briefly, 8 × 10^5^ cells were resuspended in culture medium without FBS and seeded in the upper chamber. Then the chamber was placed into a 24-well plate containing 800 μL of culture media with 20% FBS. Approximately 48 h later, the cells were fixed with paraformaldehyde and stained with crystal violet. The cells did not pass through the membrane were removed with the cotton stick while the cells that passed through the membrane were counted.

The article "miR-484 suppresses proliferation and epithelial–mesenchymal transition by targeting ZEB1 and SMAD2 in cervical cancer cells" was retracted in 2021. Reasons: duplicated images; unreliable results or conclusions; concerns about the data.

### Western blot analysis

The detailed procedures for western blot were described in a previous study [36]. The primary anti-bodies used in this study including ZEB1, SMAD2, E-cadherin, cytokeratin, vimentin, N-cadherin, fibronectin and GAPDH, which were obtained from Saier Co. (Tianjin, China). The secondary goat anti-rabbit antibodies were purchased from Sigma.

### Immunohistochemistry

The tumor tissues were fixed in 4% formaldehyde for 24 h and sent to Tangshan People’s Hospital for immunohistochemistry.

### Statistical analyses

All the data are presented as the mean ± SD. Each experiment was performed at least three times, and the analysis was performed using paired t test. p ≤ 0.05 was considered statistically significant (*p < 0.05, **p < 0.01, ***p < 0.001, ****p < 0.0001).

## Results

### miR-484 is down-regulated in cervical cancer tissues

We first examined the expression of miR-484 in 15 pairs of cervical cancer tissues and the adjacent noncancerous tissues by RT-qPCR. The results showed that miR-484 was generally down-regulated in cervical cancer tissues compared with the adjacent noncancerous tissues (Fig. 1a).

**Fig. 1:** miR-484 suppresses the proliferation of CC cells. **a** RT-qPCR showed the expression of miR-484 in 15 pairs of human cervical cancer tissues and the adjacent noncancerous tissues. U6 snRNA was used as the internal control. **b** After transfection 48 h, RT-qPCR was performed to detect miR-484 levels in HeLa or C33A cells transfected with pcDNA3/pri-miR-484 or ASO-miR-484. **c** After transfection 24, 48, 72 h, MTT assay was performed to measure cell viability in HeLa or C33A cells transfected with pcDNA3/pri-miR-484 or ASO-miR-484. **d** Colony formation assay was performed to determine the effect of miR-484 on the long-term proliferative activity of HeLa or C33A cells. The control was normalized to 1

### miR-484 inhibits cell growth of cervical cancer cells, suppresses cell cycle while exacerbates apoptosis in cervical cancer cells

First, we tested the efficiency of the plasmids pcDNA3/pri-miR-484 and ASO-miR-484 in HeLa and C33A cells with RT-qPCR. The results showed that both the plasmid and ASO-miR-484 can change the miR-484 expression efficiently (Fig. 1b). Next, MTT assays were used to test cell viability after transfecting with pcDNA3/pri-miR-484 or ASO-miR-484 at 24, 48 and 72 h. The results showed that miR-484 decreased, whereas ASO-miR-484 increased cell viability in both HeLa and C33A cells (Fig. 1c). Meanwhile, colony formation assay was performed to test the effects of miR-484 on proliferation. The results showed that the overexpression of miR-484 suppressed, whereas ASO-miR-484 increased the colony formation rate (Fig. 1d). Taken together, these results indicate that miR-484 suppresses the proliferation of HeLa and C33A cells.

The article "miR-484 suppresses proliferation and epithelial–mesenchymal transition by targeting ZEB1 and SMAD2 in cervical cancer cells" was retracted in 2021. Reasons: duplicated images; unreliable results or conclusions; concerns about the data.

To investigate the mechanisms underlying the regulation of cell growth, we examined the alterations in cell cycle progression and apoptosis caused by miR-484 in the HeLa cells using flow cytometry analysis. As shown in Fig. 2a, the overexpression of miR-484 in HeLa cells increased the percentage of cells in the G1 phase from 66.69 to 75.00% and decreased the percentage of cells in the G2/M phase from 13.8 to 7.87% (Fig. 2b). The proliferation index of the miR-484-treated cells was apparently lower than that of the negative control (Fig. 2b). In contrast, inhibition of miR-484 by antisense oligonucleotides in HeLa cells led to an increase in the percentage of cells in the G2/M phase from 13.85 to 21.90% and a decrease in the percentage of cells in the G1 phase from 65.32 to 56.87% (Fig. 2b). The proliferation index of the ASO-miR-484-treated HeLa cells was increased compared with the ASO control (Fig. 2b). In addition, flow cytometry results showed that miR-484 exacerbates apoptosis, while ASO-miR-484 inhibited apoptosis obviously in CC cells (Fig. 2c). Taken together, all these results indicated that miR-484 suppresses cell growth by both delaying the G1 to S phase and the S to G2 phase transitions and exacerbating apoptosis in CC cells.

**Fig. 2:** miR-484 suppresses cell cycle of CC cells and exacerbates apoptosis. **a**, **b** The cell cycle progression of HeLa cells was analyzed by flow cytometry. The chart shows the population of cells in G1-, S- and G2-phase (**a**) as well as the proliferation index (**b**). Proliferation index = (S + G2)/G1 (S, G2 and G1 are the percentages of cells in S-phase, G2-phase and G1-phase, respectively). **c** After transfection 24 h, apoptosis of HeLa cells was monitored by Annexin V-PI double staining and flow cytometry assay. Paclitaxel was used to induce cell apoptosis 6 h before collecting cells. The *right lower quadrant* of each plot contains early apoptotic cells, whereas the *right upper quadrant* contains late apoptotic cells. All data represent mean ± SD of three independent experiments. *p < 0.05, **p < 0.01, ***p < 0.001

The article "miR-484 suppresses proliferation and epithelial–mesenchymal transition by targeting ZEB1 and SMAD2 in cervical cancer cells" was retracted in 2021. Reasons: duplicated images; unreliable results or conclusions; concerns about the data.

### miR-484 suppresses the migration and invasion of cervical cancer cells and inhibits the EMT process

To explore the effects of miR-484 on the migration and invasion of CC cells transwell migration and invasion assays were performed. The transwell membrane was coated with Matrigel in the invasion assay. The results showed that overexpression of miR-484 significantly suppressed the migration ability by approximately 59.8 and 43.7% in HeLa and C33A cells; while blocking of miR-484 increased the migration ability by approximately 1.7- and 1.9-fold in HeLa and C33A cells respectively (Fig. 3a). The overexpression of miR-484 suppressed the invasion ability by approximately 52.1 and 44% in HeLa and C33A cells; while ASO-miR-484 increased the invasion ability by 1.6- and 1.7-fold in HeLa and C33A cells respectively (Fig. 3b).

**Fig. 3:** miR-484 suppresses the migration and invasion of CC cells and down-regulates the EMT process. **a**, **b** After transfection 48 h, cell migration (**a**) and invasion (**b**) were evaluated using a transwell system with 8 μm pores in polycarbonate membranes. Representative views of migratory or invasive cells on the membrane were presented below. All pictures were photographed at ×20 magnification. **c** Protein levels of EMT-associated markers were assessed by western blotting after transfection 48 h. **d** RT-qPCR analysis for the expression of EMT transcription factors ZEB1, Snail, Slug and Twist2 in HeLa cells transfected with miR-484 or the control vector. The control was normalized to 1. All data represent mean ± SD of three independent experiments. *p < 0.05, **p < 0.01, ***p < 0.001

It has been reported that EMT is an important mechanism correlated with migration and invasion [22]. During the transition, the expression of epithelial markers that enhance cell–cell contact decreases, while the expression of mesenchymal markers increases [17]. Therefore, we tested the expression of molecular markers to clarify the effects of miR-484 on the EMT process. As shown in Fig. 3c, the overexpression of miR-484 increased epithelial markers (E-cadherin and cytokeratin) protein levels but decreased mesenchymal markers protein levels (vimentin, N-cadherin and fibronectin) in both HeLa and C33A cells. By contrast, ASO-miR-484 decreased the epithelial markers but increased the mesenchymal markers protein levels. Importantly, RT-qPCR showed that miR-484 decreased the expression of transcription factors Snail, Slug, Twist and ZEB1 which play vital role in initiation of EMT process (Fig. 3d). With the modulation of miR-484, the expression of ZEB1 showed the greatest alteration. In summary, these results demonstrated that miR-484 suppresses the migration and invasion and inhibits the EMT process of CC cells.

The article "miR-484 suppresses proliferation and epithelial–mesenchymal transition by targeting ZEB1 and SMAD2 in cervical cancer cells" was retracted in 2021. Reasons: duplicated images; unreliable results or conclusions; concerns about the data.

### miR-484 targets and down regulates ZEB1 and SMAD2 expression

As miR-484 suppresses cervical cancer cell growth, migration, and invasion, it is important to understand which targets are directly responsible for the observed phenotypes. We used three prediction algorithms (TargetScan, miRecords, and PITA) to predict the targets for miR-484 in common. There were 258 candidate targets shared by all the three databases (the overlapping fraction), in which only four genes involved in the regulation of EMT process (Fig. 4a). Based on our data (Fig. 3d) and previous reports, we chose ZEB1 and SMAD2 for further study. ZEB1 usually acts as a key transcription factor which can induce EMT, and our data had shown ZEB1 expression was altered with the modulation of miR-484 (Fig. 3d), which suggested that ZEB1 may be a bona fide target of miR-484. Moreover, the previous work in our lab has demonstrated that SMAD2 promotes cell growth, migration, invasion, and EMT in Human CC Cell Lines [6]. Other reports have revealed that Smads interact with the ZEB promoter [30, 31]. Therefore, we chose SMAD2 as a second candidate target of miR-484.

**Fig. 4:** miR-484 directly targets SMAD2/ZEB1 and down-regulates their expressions. **a** The venn diagram shows the potential target genes (overlapping fraction) that were shared by all three databases. **b** The predicted binding sites for miR-484 in the 3′UTR of SMAD2 and ZEB1 and the mutations in the binding sites are shown. **c** The EGFP reporter assay was performed in HeLa or C33A cells co-transfected with pcDNA3/EGFP-SMAD2/ZEB1 3′UTR wild type or pcDNA3/EGFP-SMAD2/ZEB1 3′UTRmut with pri-miR-484 or ASO-miR-484. The fluorescence intensities were measured at 48 h after transfection. **d** Western blot assays were used to detect the SMAD2 and ZEB1 protein levels in HeLa or C33A cells transfected with pcDNA3/pri-miR-484, ASO-miR-484 or their corresponding controls. **e** Western blot assays tested the effect of SMAD2 on the expression of ZEB1. *p < 0.05, **p < 0.01, ***p < 0.001, ns, no significance. All the *bars* indicate the means ± SDs. All experiments were performed at least triplicates

To confirm whether SMAD2 and ZEB1 are direct targets of miR-484 in human CC cells, we used an EGFP reporter system, in which we cloned the wild SMAD2/ZEB1 3′-UTR or a mutant SMAD2/ZEB1 3′-UTR downstream of the EGFP reporter gene (Fig. 4b). Co-transfection was performed with an RFP reporter as a transfection normalizer and with either pri-miR-484 or ASO-miR-484 in HeLa cells. After 48 h, we determined the fluorescence intensity. As shown in Fig. 4c, overexpression of miR-484 decreased the fluorescent intensity of the wild type ZEB1/SMAD2 3′UTR. In contrast, ASO-miR-484 increased the fluorescent intensity (Fig. 4c). However, neither the over-expression nor inhibition of miR-484 affected the fluorescent intensity of the mutant ZEB1/SMAD2 3′UTR (Fig. 4c).

The article "miR-484 suppresses proliferation and epithelial–mesenchymal transition by targeting ZEB1 and SMAD2 in cervical cancer cells" was retracted in 2021. Reasons: duplicated images; unreliable results or conclusions; concerns about the data.

We also explored the functions of miR-484 in the expression of endogenous ZEB1/SMAD2 protein by western blot. The results showed that the overexpression of miR-484 decreased, while ASO-miR-484 increased the expression of ZEB1/SMAD2 (Fig. 4d). Thus, the results demonstrate that miR-484 directly targets the 3′UTR of ZEB1/SMAD2 and down-regulates their protein expressions in CC cells.

Interestingly, we observed that overexpression of SMAD2 led to an increase in ZEB1 protein level (Fig. 4e). Conversely, decreased SMAD2 prevented up-regulation of ZEB1 protein level. This indicates that SMAD2 is an upstream regulator of ZEB1 and regulated its expression. These results demonstrate that miR-484 directly targets the 3′UTR of ZEB1 and SMAD2 mRNA and down-regulates their expression simultaneously.

### ZEB1 and SMAD2 rescue the suppression of the malignant behavior induced by miR-484

Based on our results, we questioned whether the effect of miR-484 on CC cells is mediated by its down-regulatory effect on SMAD2 and ZEB1 expression. We performed rescue experiments to address this issue. First, we co-transfected miR-484 with the SMAD2/ZEB1 expression plasmid without the 3′UTR which has been proved worked (Fig. 5a) and confirmed the over-expression of SMAD2/ZEB1 could rescue the decrease in SMAD2/ZEB1 protein levels caused by miR-484 (Fig. 5a). Then we performed a series of functional rescue experiments. As expected, the restoration of SMAD2/ZEB1 expression mostly blocked the inhibitory effects of miR-484 on the cell viability (Fig. 5b), colony formation rate (Fig. 5c) and cell cycle (Fig. 6a). SMAD2/ZEB1 also restored the apoptosis induced by miR-484 (Fig. 6b). In addition, the restoration of SMAD2/ZEB1 can also counteract the suppression of the migration/invasion via miR-484 (Fig. 7a, b). Meanwhile, the ectopic expression of SMAD2/ZEB1 counteracts the inhibition of EMT induced by miR-484 in CC cells (Fig. 7c).

**Fig. 5:** The ectopic expression of SMAD2 and ZEB1 counteracts the inhibition of cell proliferation induced by miR-484. **a** CC cells were co-transfected with pcDNA3/pri-miR-484 and pFlag-SMAD2/ZEB1 without its 3′UTR or the control vector and western bolt assay was used to determine the restoration of SMAD2 or ZEB1 protein levels by pFlag-SMAD2/ZEB1 in the presence of miR-484. **b** After transfection 48 h, MTT assay was performed to detect cell viability in CC cells. **c** The transfected cells were submitted to colony formation assays to test the proliferation of CC cells. All data represent mean ± SD of three independent experiments. *p < 0.05, **p < 0.01, ***p < 0.001

**Fig. 6:** The ectopic expression of SMAD2 and ZEB1 counteracts the inhibition of cell cycle and the promotion of apoptosis induced by miR-484. **a** The cell cycle progression of HeLa cells was analyzed by flow cytometry. **b** After transfection 24 h, apoptosis of HeLa cells was monitored by Annexin V-PI double staining and flow cytometry analysis. All data represent mean ± SD of three independent experiments. *p < 0.05, **p < 0.01, ***p < 0.001

**Fig. 7:** The ectopic expression of SMAD2 and ZEB1 counteracts the inhibition of migration, invasion and EMT progression induced by miR-484. **a**, **b** Transwell migration/invasion assays and three-dimensional Matrigel culture to test the cells’ abilities to migration (**a**) and invasion (**b**). **c** Protein levels of EMT-associated markers were assessed by western blotting after transfection for 48 h. *p < 0.05, **p < 0.01, ***p < 0.001. All the *bars* indicate the means ± SDs. All experiments were repeated at least three times

To confirm the deduce that the effect of miR-484 on CC cells is mediated by its down-regulatory effect on SMAD2 and ZEB1 expression in an inverse way, ASO-miR-484 along with pshR-ZEB1/SMAD2 was co-transfected into HeLa and C33A cells. As anticipated, the effects of miR-484 blocking on cell growth were significantly impaired when ZEB1/SMAD2 was suppressed (Fig. 8a, b). Furthermore, the expressions of EMT markers in the miR-484-blocking cells were restored to the normal levels after knocking-down of ZEB1/SMAD2 (Fig. 8c). In conclusion, all these data indicate that SMAD2 and ZEB1 are functional targets of miR-484 in cervical cancer cells.

The article "miR-484 suppresses proliferation and epithelial–mesenchymal transition by targeting ZEB1 and SMAD2 in cervical cancer cells" was retracted in 2021. Reasons: duplicated images; unreliable results or conclusions; concerns about the data.

**Fig. 8:** Knockdown of SMAD2/ZEB1 abrogates the effects induced by ASO-miR-484. **a** After co-transfection with ASO-miR-484 and pshR-SMAD2/ZEB1 or the control vector for 48 h, MTT assay was performed to detect cell viability in CC cells. **b** The transfected cells were submitted to colony formation assays to test the proliferation of CC cells. **c** The expression of EMT markers (E-cadherin and vimentin) was detected by western blot analysis. All data represent mean ± SD of three independent experiments. *p < 0.05, **p < 0.01, ***p < 0.001

### miR-484 is inversely correlated with SMAD2 and ZEB1 expressions in cervical cancer tissues and cell lines

To further explore the expression levels of ZEB1 and SMAD2 in cervical cancer, we performed RT-qPCR analyses to examine their expression levels in 15 pairs of CC tissues and adjacent non-tumor tissues as well as a panel of cervical cancer cell lines. We found that ZEB1 and SMAD2 were both upregulated in cancer tissues compared with the adjacent non-tumor tissues, which was opposite to the expression pattern of miR-484 (Fig. 9a). By Pearson’s correlation analysis, miR-484 presented a reverse correlation with the expression of ZEB1 (r = −0.70, p < 0.01) and SMAD2 mRNA (r = −0.65, p < 0.001) (Fig. 9b). Interestly, the expression of ZEB1 and SMAD2 presented a positive correlation (r = 0.61, p < 0.05) (Fig. 9b). We also performed immunohistochemistry (IHC) to determine the expressions of ZEB1 and SMAD2 in clinical cervical samples. The results further demonstrated that ZEB1 and SMAD2 were both upregulated in cervical cancer tissues compared with the normal cervix (Fig. 9e).

**Fig. 9:** The inverse correlation between the expression of miR-484 and ZEB1/SMAD2 in cervical cancer tissues and cell lines. **a** RT-qPCR showing the expression of SMAD2 and ZEB1 in 15 pairs of human cervical cancer tissues and the adjacent noncancerous tissues. U6 snRNA was used as the internal control. **b** Pearson’s correlation analysis indicated the negative correlation between the expression of miR-484 and ZEB1 (r = −0.55*) and SMAD2 (r = −0.65***). **c** RT-qPCR showing the expression of miR-484, SMAD2 and ZEB1 in cervical cancer cell lines compared with NCx. U6 snRNA and β-actin were used as the internal controls. **d** Western blot were used to detect the ZEB1 and SMAD2 protein levels in cervical cancer cell lines compared with NCx. All data represent mean ± SD of three independent experiments. *p < 0.05, **p < 0.01, ***p < 0.001, ****p < 0.0001. **e** Representative IHC images showing the expression level of SMAD2 and ZEB1 in cervical cancer and normal cervix (×20)

We also determined the expressions of miR-484, ZEB1 and SMAD2 using RT-qPCR and western blotting analyses in a panel of cervical cancer cell lines as well as normal cervical keratinocytes cells. RT-qPCR and western blotting analyses revealed a significant inverse correlation between miR-484 and ZEB1/SMAD2 expression levels in different cervical cancer cell lines (Fig. 9c, d). The expression of ZEB1/SMAD2 in HeLa cells changed the most sharply while in C33A cells changed the least sharply compared with others. The expression of miR-484 and SMAD2/ZEB1 in both the tissues and cell lines indicated that miR-484 had reverse correlation with SMAD2/ZEB1, and that SMAD2 and ZEB1 had positive correlation with each other.

In conclusion, miR-484 regulated cell proliferation and EMT process through both directly and indirectly targeting ZEB1. As shown in Fig. 9e, we illustrated the regulation network reported by this work. To our notice, ZEB1 was the central molecules in this regulatory pathway. On one hand, miR-484 could inhibit cell proliferation and EMT process by directly targeting ZEB1. On the other hand, miR-484 suppresses cell growth and EMT by directly targeting SMAD2, an important upstream regulator of ZEB1 (Fig. 10). These results indicate that miR-484 exerts multiple pathways of regulation on ZEB1 expression resulting in the inhibition of cell growth and EMT.

The article "miR-484 suppresses proliferation and epithelial–mesenchymal transition by targeting ZEB1 and SMAD2 in cervical cancer cells" was retracted in 2021. Reasons: duplicated images; unreliable results or conclusions; concerns about the data.

**Fig. 10:** Schematic that describes the role of miR-484 in CC cells. miR-484 regulated proliferation and EMT process through both directly and indirectly targeting ZEB1 in CC cells

## Discussion

miRNAs have been indicated to be important regulators of a variety of biological processes, and their aberrant expressions are relevant to cancer initiation and development. In recent years, miRNAs were reported as potential biomarkers as therapeutic approaches in human cancers [37]. Understanding the role of miRNAs in cervical cancer will provide theoretical basis for miRNA-specific personalized treatment and molecular-targeted therapy.

miR-484 was originally discovered to be associated with resistance to chemotherapeutic agents in cancer [38]. This year, an aberrant expression of miR-484 has also been described in high-fat-diet-induced tumours, with a fluctuant miR-484 overexpression during feeding [39]. Ectopic expression of miR-484 initiates tumourigenesis and cell malignant transformation of HCC through synergistic activation of the TGF-β/Gli and NF-κB/IFN-I pathways [14]. This indicated that miR-484 may act as a significant role in tumor metastasis including EMT process. To our understanding, the functional study of miR-484 in cervical cancer is still missing. Here, we demonstrated that miR-484 was down-regulated in cervical cancer tissues compared to adjacent non-tumor tissues, which is different from the result in HCC. These differences may be due to the different types of cancer and the phases of the cancer, but the mechanisms need to be elucidated in the future. For example, miR-200s is downregulated and inhibit local invasion in breast cancer but enhances spontaneous metastasis and colonization of lung adenocarcinoma [40]. Functional analyses revealed that overexpression of miR-484 suppressed the malignant behavior of cervical cancer cells. Specifically, miR-484 overexpression significantly inhibited the cell proliferation, migration, invasion and EMT, whereas ASO-miR-484 enhanced these oncogenic features. In addition, western blot indicated that the expression of EMT markers including E-cadherin, cytokeratin, vimentin, N-cadherin and fibronectin were significantly modulated by miR-484, which is consistent with the formation of EMT. Collectively, miR-484 functions as a tumor suppressor in cervical cancer cells.

miRNAs generally play their roles by regulating their target genes. To better understanding the role of miR-484 in CC, we applied bioinformatics analyses to predict that the 3′UTR of SMAD2/ZEB1 contains miR-484 binding sites. EGFP reporter assay demonstrated that miR-484 directly targets SMAD2 and ZEB1 transcripts. Western blot analyses showed the decreased expression of ZEB1 and SMAD2 upon overexpression of miR-484 and vise versa. Functionally, overexpression of miR-484 could inhibit cell proliferation, migration, invasion and EMT, while the ectopic expression of SMAD2/ZEB1 abrogated the inhibitory effects of miR-484 on these tumorigenic features in cervical cancer cells. Meanwhile, we also showed that knocking-down of SMAD2/ZEB1 abrogated the tumorigenic effects induced by ASO-miR-484. Thus, we concluded that miR-484 may function as tumor suppressor by down-regulation of ZEB1 and SMAD2 expressions in cervical cancer.

The article "miR-484 suppresses proliferation and epithelial–mesenchymal transition by targeting ZEB1 and SMAD2 in cervical cancer cells" was retracted in 2021. Reasons: duplicated images; unreliable results or conclusions; concerns about the data.

Upregulation of the expression of ZEB1 plays an important role in the progression and metastasis in many cancers [24–26], including cervical cancer [27]. Our previous study has shown that SMAD2 promotes cell growth by facilitating the G1/S phase transition, enhances cell migration and invasion through regulated EMT in CC cell lines [6]. In addition, regulating SMAD2 by miRNAs has been identified to be involved in the TGFβ-induced EMT. For example, miR-18b targets SMAD2 and inhibits TGF-β1-induced differentiation of hair follicle stem cells into smooth muscle cells [41], and miR-27a inhibits colorectal carcinogenesis and progression [42]. Expectedly, ectopic expression of SMAD2 counteracts the inhibition of EMT induced by miR-484 in CC cells. The restoration of SMAD2/ZEB1 expression mostly blocked the inhibitory influence of miR-484 on malignant behavior (Figs. 5, 6, 7). The expression of miR-484 and SMAD2/ZEB1 in the tissues and cell lines demonstrated that miR-484 had negative correlation with SMAD2/ZEB1, and that SMAD2 had positive correlation with ZEB1 (Fig. 9b, c). This result further supported that SMAD2 is an upstream protein of ZEB1 and they are both regulated by miR-484. Previous work has demonstrated that SMAD directly binds to the promoter of the ZEB factor and indirectly regulates EMT [30, 31], which is in accordance with our results in CC. In summary, all these results prove that miR-484 inhibits the development of CC and may partially (if not completely) through down-regulating SMAD2 and ZEB1 expressions.

Except for ZEB, other transcription factors such as Snail, Slug and Twist are also the master regulators of EMT [22], which can activated by TGFβ directly and repress the transcription of E-cadherin [23]. The TGFβ/ZEB/miR-200 double-negative feedback loop has been found and postulated to explain both the stability and interchangeability of the epithelial versus mesenchymal phenotypes in MDCK cell systems [43, 44]. In the present study, we found that miR-484 could target both SMAD2 and ZEB1 genes simultaneously, and ZEB1 is regulated by SMAD2 as well, which is different from The ZEB/miR-200 double-negative feedback loop. Interesting, our results also showed that miR-484 affects the expression of Snail, Slug and Twist as well, which may due to miR-484 regulating ZEB1 to the EMT-related regulators, while the detailed regulatory mechanism need to be further investigated. These results indicate that miR-484 exerts multiple pathways of regulation on EMT and highlight the importance of stringently regulating transcription factors. These findings also fit the emerging concept that miRNAs fine-tune gene expression to precisely modulate essential biological processes and provide a mechanistic view of miRNA-based regulation on specific molecules and markers involved in cancer metastasis.

The article "miR-484 suppresses proliferation and epithelial–mesenchymal transition by targeting ZEB1 and SMAD2 in cervical cancer cells" was retracted in 2021. Reasons: duplicated images; unreliable results or conclusions; concerns about the data.

Despite these studies, further development of the underlying mechanisms need to be investigated. And our next work is to found out the upstream regulatory mechanisms of miR-484 in CC cells.

## Conclusions

In summary, our study demonstrated that miR-484 plays an important role in tumorigenesis and related to the EMT process in CC for the first time. miR-484 inhibits the proliferation, and exacerbates apoptosis, suppresses migration, invasion and EMT process through the down-regulation of ZEB1 and SMAD2 expression and functions as a tumor suppressor gene. In other words, miR-484 regulated EMT process through both directly and indirectly targeting ZEB1. Altogether, our findings provide new insights into the roles of miR-484 in cervical carcinogenesis and imply its potential applications as new biomarkers in cervical cancer.

## Abbreviations

miRNAs: microRNAs
CC: cervical cancer
NCx: normal cervical keratinocytes
EMT: epithelial–mesenchymal transition
ZEB: zinc finger E-box-binding homeobox
ASO-miR-484: the 2′-*O*-methyl-modified antisense oligonucleotide of miR-484
ASO-NC: the scramble control oligonucleotides
MTT: the 3-(4,5-dimethylthiazol-2-yl)-2,5-diphenyl-tetrazolium bromide
